# Study protocol for a randomized controlled pilot-trial on the semiocclusive treatment of fingertip amputation injuries using a novel finger cap

**DOI:** 10.1097/MD.0000000000008224

**Published:** 2017-10-13

**Authors:** Jurek Schultz, Susann Leupold, Xina Grählert, Roland Pfeiffer, Uta Schwanebeck, Percy Schröttner, Barbara Djawid, Wladislav Artsimovich, Karol Kozak, Guido Fitze

**Affiliations:** a Pediatric Surgery; b Coordinating Centre for Clinical Trials Dresden; c Institute of Medical Microbiology and Hygiene, Carl Gustav Carus Medical Faculty, Technische Universität Dresden, Fetscherstrasse; d Fraunhofer Institute for Material and Beam Technology IWS Dresden; e Carl Gustav Carus Medical Faculty, Technische Universität Dresden, Fetscherstrasse, Dresden, Germany; f Wrocław Medical University, Wybrzeże Ludwika Pasteura 1, Wrocław, Poland.

**Keywords:** fingertip injuries, hand surgery, pediatric surgery, RCT, regeneration, semiocclusive dressing

## Abstract

**Introduction:**

Fingertip amputation injuries are common in all ages. Conservatively treated fingertips can regenerate skin and soft tissues to form a functionally and cosmetically excellent new fingertip. Little is known about this ability that, in humans, is confined to the fingertips. Even less is known about the role of the bacteria that regularly colonize these wounds without negative impact on regeneration and healing.

As an alternative to surgery, self-adhesive film dressings are commonly used to establish a wet chamber around the injury. These dressings leak malodorous wound fluid eventually until the wound is dry. Having that into consideration, we have therefore developed a silicone finger cap that forms a mechanically protected, wet chamber around the injury for optimal regeneration conditions. It contains a puncturable reservoir for excess wound fluid, which can be thus routinely analyzed for diagnostic and research purposes.

This study protocol explains the first randomized controlled trial (RCT) on the semiocclusive treatment of fingertip amputations in both children and adults comparing traditional film dressings with the novel silicone finger cap. Being the first RCT using 2 medical devices not yet certified for this indication, it will gather valuable information for the understanding of fingertip regeneration and the design of future definitive studies.

**Methods and analysis:**

By employing an innovative pseudo-cross-over-design with a dichotomous primary endpoint based on patients preference, this pilot study will gain statistically significant data with a very limited sample size. Our RCT will investigate acceptance, safety, effectiveness, and efficacy of this novel medical device while gathering information on the clinical course and outcome of conservatively treated fingertip injuries. A total of 22 patients older than 2 years will be randomly assigned to start the conservative treatment with either the traditional film-dressing or the novel finger cap. The treatment will be changed to the other alternative for another 2 weeks before the patient or the guardian is confronted with the decision of which method they would prefer for the rest of the treatment (if required).

**Ethics and dissemination:**

Ethical approval (EK 148042015) of the study protocol has been obtained from Institutional Review Board at the TU Dresden. The trial is registered at the European Database on Medical Devices (EUDAMED-No.: CIV-15-03-013246) and at ClinicalTrials.gov (NCT03089060).

## 1 Introduction

Fingertip injuries are very common. In pediatric emergency departments, fingertip injuries account for up to 2%^[1]^ of appearances of children under 14 years of age with 25% of these injuries being more serious, needing surgical treatment, in 15% of the cases under general anesthetics.^[1]^

Already in 1974, Illingworth reported on pediatric fingertip injuries with substance loss, that were treated conservatively with very good success.^[2]^ The superiority of the conservative approach was afterwards demonstrated in comparative studies.^[2–5]^ Later, sulphadiazine gloves, and thus a method of occlusive dressing that formed a wet chamber around the injury, were used.^[6]^ Söderberg et al^[7]^ used ink tattoos on the wound edge to show that human fingertips regenerate de novo under conservative treatment. Additionally, the use of film dressings to occlude the injured fingertips was demonstrated in a series of 200 patients in 1993.^[8]^ The authors concluded that this kind of treatment should be recommended for all fingertip injuries.^[8]^

Surgical approaches for fingertip amputation injuries that cannot be subjected to primary closure include stump plasties, local, or distant flaps (eg, V-Y-plasty, etc), microsurgical replantation, composite grafts, or skin transplants.^[9]^ There are only little and conflicting data on the indication of conservative versus surgical techniques. Controversies also exist on necessary wound disinfection, if exposed bone should be shortened before any occlusive dressing is applied and, whether or not, amputates should be reattached as composite grafts.^[10–12]^

In many centers the conservative management of fingertip injuries is accomplished with self-adhesive film dressings.^[8,13]^ However, this management is sometimes difficult, especially since these dressings do not stick to wet skin. Conventional dressings do not form a protected chamber around the wound, additional splinting is often needed^[5,6]^ and leakage of malodorous wound fluid is very disturbing. Therefore, we have optimized the conventional occlusive dressings by applying techniques known from silicone finger ortheses and designed a novel silicone finger cap that deals with the aforementioned issues.

This novel silicone finger cap is now evaluated for the first time in an investigator initiated, randomized controlled clinical trial regarding the acceptance of the finger cap in comparison to conventional film dressings using a pseudo-cross-over study design. As both medical devices are not certified for the treatment of deeper wounds and exposed bone, this randomized controlled trial (RCT) is a pilot study by definition. By employing a pseudo-cross-over-design with a summative dichotomous primary end-point (patient preference) we will gain statistically significant data despite the limited sample size while gathering important data with a variety of secondary end-points to plan for future definitive studies and better understand fingertip regeneration.

As well as evaluating the safety and efficacy of this novel treatment, secondary endpoints of our study include clinical, functional, microbiological, and quality-of-life parameters. Additionally, our RCT includes a substudy for the harvesting of wound fluids from the puncturable reservoir incorporated in our finger cap. This will allow the search for human and bacterial soluble factors that may promote tissue regeneration and limit bacterial growth to local colonization. Our study starts enrolling patients in August 2017.

## 2 Methods and analysis

### 2.1 Study design

This pilot study is a monocentric, prospective, randomized, controlled clinical trial. Primarily, it will investigate the acceptance of the silicone finger cap in comparison to conventional film dressings. Using sealed neutral envelopes prepared by external staff from the Coordinating Centre for Clinical Trials, our patients will be randomly assigned by the study doctors to begin their treatment either with the finger cap or the film dressing. After 2 weeks they will be changed to the other treatment modality. After another 2 weeks have passed, patients/guardians will have to decide prior to the dressing change which treatment they would like to receive thereafter if further occlusion is needed. The primary clinical endpoint of this pseudo-cross-over study (Fig. 1) is the rate of patients/guardians who decide to continue their treatment with the silicone finger cap. Further secondary endpoints include the determination of the safety of the finger cap in comparison to the film dressing and the determination of disease-specific quality of life during the treatment with the silicone finger cap in comparison to the film dressing using a modified quality of life Wuerzburg Wound Score regarding pain during application and treatment with the finger cap, restrictions in daily activities and quality of life.^[14]^ Also the necessity of unplanned dressing changes in comparison to the film dressing and changes in microbiological colonization in the wound during the treatment will be registered. Additionally, we will measure the reepithelialization rate and determine the tissue growth at 28 days and at 4 months after the injury. We will also test the function of the regenerated perspiratory glands and the clinical outcome in terms of sensitivity and motility of the injured fingertip as well as cosmetic aspects.

**Figure 1:** Pseudo-cross-over study design of this study.

### 2.2 Treatment group

The silicone finger cap consists of a thin and soft silicone shaft that surrounds the basis of the finger and provides the semiocclusive seal without the need for additional adhesives. It is thus a further development of conventional occlusive means such as self-adhesive films or fingers of sterile rubber gloves. The finger cap forms a protected chamber of more rigid silicone around the distal phalanx that is close to the original, anatomical form, and size of the fingertip. The more rigid silicone is continued in a narrow bar all the way to the base of the finger cap thus splinting the injured finger enough to care for undisturbed healing while allowing some movement in all finger joints. A reservoir for excess wound fluid is connected to the wound chamber by capillaries, thus enabling free diffusion in between the wound and the reservoir (Fig. 2). This reservoir can be punctured with a regular injection needle. The used medical silicone Dragon Skin Series Part A&B (KauPo, Spaichingen, Germany), Silastic Q7-4720 Biomedical Grade ETR Elastomer and Silastic Q7-4765 Biomedical Grade ETR Elastomer (Dow Corning, Midland, TX) is permeable to oxygen to some extent but impermeable to water vapor. For this series all finger caps are individually handcrafted by Orthopedic and Rehabilitation Engineering Dresden (GmbH), Dresden, Germany, the sponsor of this clinical trial. Besides, the sponsor office was committed to the Coordinating Centre for Clinical Trials Dresden.

**Figure 2:** Novel silicone finger cap. (A) dorsal view, (B) sagittal view: (1) apex, (2) protective cap of rigid silicone, (3) reservoir, (4) capillary, (5) chamber for injured finger, (6) thin and soft silicone, (7) incorporated splint of more rigid silicone, and (8) base.

### 2.3 Control group

In our control group, we start the treatment with a self-adhesive polyurethane film dressing as it is used in most centers as standard therapy.^[4,8,13,15–18]^ Opsite Flexigrid transparent dressing (Smith & Nephew Medical Limited, Hull, England) is a transparent film dressing, comprised of a polyurethane film with acrylic adhesive. It is Communauté Européenne (certification mark indicating conformity with European legislation)-certified and it is classified according to the European classification of medical devices in group IIa.

### 2.4 Inclusion and exclusion criteria

The participants are recruited by trained surgeons in the Emergency Department of the University Hospital Carl Gustav Carus at the Technische Universität Dresden, Germany. We include male and female patients older than 2 years with full skin substance defects distal to the distal interphalangeal joint unsuitable for primary surgical closure without further substance loss. No more than 5 fingers per patient may be injured. Patients must have a circumference of the proximal phalanx in between 3.0 and 9.0 cm. In addition, a signed written informed consent must exist.

We exclude the participation of any patient with known hypersensitivity against medical silicone or self-adhesive films. Further exclusion criteria are bony injuries requiring a surgical intervention, bite injuries, or chronic dermatological disorders of the hand. Furthermore, intake of medications affecting wound healing, such as systemic (noninhalative) glucocorticoids, immunosuppressive, or blood-thinning medications are exclusion criteria. Patients with a known wound healing disorder are also excluded from this clinical trial. In addition, ongoing or recently finished chemotherapy, immunodeficiencies or diabetes mellitus, are exclusion criteria. In accordance to §20 of the German Medical Device Act, pregnant or breastfeeding women, as well as any women, when a pregnancy at the beginning or during the course of the study cannot be ruled out (ie, not postmenopausal, no bi-lateral oophorectomy or hysterectomy, no contraceptive method with pearl index less than 1%, no sexual abstinence, or partner with vasectomy) will have to be excluded. Beyond that, patients who are suffering from an addiction or other diseases, which do not allow them to assess the entity, scope, and possible consequences of this clinical trial are also excluded. The same applies for patients who are not cooperative or who already participated in other clinical trials within the last 4 weeks.

### 2.5 Procedure

Screening, recruitment, and treatment of our patients take place in our emergency department. Initially, the patient's medical history along with the accident history is obtained. All patients with fingertip amputations who present themselves to the emergency department are informed about this clinical trial. The injury is examined and the inclusion respectively exclusion criteria are checked. We routinely perform an X-ray examination to exclude bony injuries. Additionally women of childbearing age have to provide a pregnancy test prior to that. In case all inclusion and no exclusion criteria are fulfilled patients get comprehensively informed about the clinical trial and the informed consent is obtained by the trained surgeon. Randomization takes place through prepared nontransparent and consecutively numbered envelops and determines the initial treatment group (conventional film dressing or silicone finger cap). Afterwards, the respective occlusive dressing is applied according to the randomization result. We check the dressing 1 day after initial application for correct fitting. Afterwards we conduct clinical controls weekly to check for correct fitting of the occlusive dressing, to enquire possible adverse events and serious adverse events, and to take photos of the dressing and possibly of the wound. In case, the patient has got a silicone finger cap we aspirate wound fluid out of the reservoir to examine the microbiological colonization of the wound. If the patient has got an occlusive film dressing, no microbiological examination can be performed except for an initial smear and a 2nd smear when the film dressing is removed after 2 weeks. As a substudy of this clinical trial, excess wound fluid that is not used for microbiological analyses is preserved at −80 °C for future proteome analyses. Furthermore, patients are asked to complete a modified quality of life Wuerzburg Wound Score at each of their visits.

On day 14 after the injury, the occlusive dressing method is changed. Patients treated with the conventional film dressing get a silicone finger cap and vice versa. Further 14 days later the patient decides which dressing she or he respectively the guardians would prefer for the remaining treatment if needed before the dressing is removed. The chosen treatment is then applied if further treatment is needed. At day 42 after the injury the treatment of the wound is orderly finished and the wound should be reepithelialized. The occlusive dressing is removed and photographs of the injury site are taken. If the wound is not fully epithelialized at this point, a conventional film dressing is used as long as further occlusion is needed. Final follow-up examination takes place 4 months after the injury. At the follow-up we test the function of the perspiratory glands and the regeneration of the fingerprint using Moberg Ninhydrin test.^[19]^ Also the range of motion in the distal interphalangeal, proximal interphalangeal and metacarpophalangeal joints, and the 2-point-discrimination threshold in the area of the injury is checked in comparison to the corresponding finger of the contralateral hand.^[20]^ Moreover, we also measure the soft tissue thickness above the bone in the region of the healed injury using medical ultrasound. Finally, patients have to complete a follow-up questionnaire. At each visit the dressing or, when applicable, the exposed finger is photographed from all perspectives. High definition photographs will be digitally analyzed and kept for documentation purposes. In this study, we will introduce a new volume-rendering method for monitoring finger growth 3-dimensionally. Photographs will be rendered in 3-dimensional models and advanced 3-dimensional segmentation, and filtering algorithms will be used to measure volume progress of the injured finger. This method will allow monitoring of tissue recovery in micrometers quality.

### 2.6 Statistics

#### 2.6.1 Proposed sample size

There is no certified medical device available for the conservative management of fingertip amputation injuries. Opsite Flexigrid (Smith & Nephew Medical Limited, Hull, England) has not been certified for full thickness amputations injuries as described, and our novel finger cap has never been used before in a controlled trial. Therefore, this study is per definition a pilot study that has to be limited to a small sample size in order to comply to German and European legislation as well as to guidelines of good clinical practice.

The primary objective is the rate of patients who decide for the silicone finger cap at day 28. At this point they have experienced both methods (conventional film dressings and silicone finger cap) for 2 weeks each. This rate can be regarded as a measure of the acceptance of the silicone finger cap. If 80% of the patients in this study decide for the silicone finger cap we consider the hypothesized superiority of the finger cap as verified. Assuming that approximately 80% of the patients decide for the silicone finger cap, 20 patients (95% confidence interval, one-sided, 65% lower limit, the distance from the rate to the lower limit of the confidence interval is at most 15%) are needed (Program nQuery-Advisor 6.01, Copyright^©^ 1995–2005, Janet D Elashoff). When considering 2 possible drop-outs, 22 patients must be included.

### 2.7 Randomization

Based on a computer-generated randomization list (nQuery Advisor 6.01, Janet D. Elashoff), opaque, numbered envelops are produced at the Coordinating Centre for Clinical Trials. These envelopes contain the randomization result with the assignment to treatment group A or B (see Fig. 1). They are opened in ascending order after the consent of the patient/guardian has been obtained. The study doctor must note the patient identification number and the date and time of the randomization and confirm by his signature.

### 2.8 Statistical analysis

A list of imaginable complications and risks with possible management plans is part of the study protocol. In case of changes in the treatment due to complications or patient requests, patients can be treated accordingly in our clinic. All randomized patients who will be treated with the silicone finger cap or the film dressing will be included in the intent-to-treat-analyses.

The primary objective of the study is to verify the hypothesis that the silicone finger cap is superior to the conventional film dressing in regards to its acceptance by the patients/guardians. The primary endpoint is the rate of patients who decide up to day 28 to continue their treatment with the silicone finger cap. If this rate is at least 80% and the lower limit of the confidence interval is not less than 65%, the silicone finger cap is considered to be much better accepted than the conventional method.

The secondary target parameters are exploratively evaluated. Secondary endpoints are analyzed according to their scale level: for steady endpoints, mean and standard deviation, or medians and quartiles (graphically corresponding to confidence intervals or boxplots), for the categorical endpoints absolute and appropriate relative frequencies are used. Depending on the distribution of the variables to be analyzed the *t* test, the *U* test and the Chi test^[2]^ are used. For paired comparisons, the paired *t* test is used in the case of normally and the Wilcoxon test in the case of nonnormally distributed variables. Sub-group analyses according to patient age, injury severity, and mechanism of injury will be performed if possible. The statistical analysis is carried out using the SPSS program system (International Business Machines Corp. New Orchard Road, Armonk, NY) and the SAS System (SAS Institute Inc., 100 SAS Campus Drive, Cary, NC) for Windows program in the currently available versions.

### 2.9 Data management

All efforts will be made to avoid missing data, especially for the main target criteria. If a patient discontinues the trial, but a final visit was done, the data of this visit will be used for calculation of the main target criteria. The specific dealing of missing data will be determined in a data review meeting before starting statistical analyses.

All relevant patient data and test results have to be documented as soon as possible in an electronical Case Report Form (eCRF) and have to match with the source data. Source data will be verified by clinical monitoring according to the monitoring manual. Missing data or deviations will be justified and corrected only by authorized persons. Changes and corrections will be documented with an audit trail of the trial software.

All data that will be excluded before the first application of the investigational product or its reference product also have to be documented in the eCRF.

Data entry, maintenance, and handling will be done according to good clinical practice with the trial software MACRO 4 (InferMed Ltd, London, UK). There will be a validation of the data with programmed validity and consistency checks by the trial software. After finishing the investigation, the entry of all relevant data, and the clarification of all queries, the data base will be closed. After these procedures are completed, the data will be released for statistical analyses.

### 2.10 Monitoring

Because of the low case number a data review committee and interim analyses are not planned. However, a risk-based monitoring is performed by the Coordinating Centre for Clinical Trials Dresden according to DIN EN ISO 14155:2012-01 and national regulations.

Additionally, every adverse effect or product deficiency is part of the study documentation. Adverse effects have to be documented in the eCRF. Product deficiencies will be reported directly to the sponsor. Severe adverse events will be reported according to the regulatory requirements.

### 2.11 Ethics and dissemination

This study was approved by the German Federal Institute for Drugs and Medical Devices to be conducted in compliance with §22a Act on Medical Devices (AZ 94.1.05-5660-10348). Besides, this study was approved by the Ethics Committee of the Technische Universität Dresden (EK 148042015). Furthermore, the trial is registered at the European Database on Medical Devices (EUDAMED-No.: CIV-15-03-013246) and at ClinicalTrials.gov (NCT03089060; registration date: March 17, 2017).

Participants will be insured with Chubb Insurance Company of Europe SE for up to €500.000 per participant to cover for any harms caused by the participation in this trial.

Trial results will be disseminated through scientific conference presentations and by publication in scientific journals. Modifications of the trial protocol will only be done in consultation with investigators and the sponsor. Substantial amendments of the protocol require the approval of the Ethics Committee and the national authority (German Federal Institute for Drugs and Medical Devices).

## Acknowledgments

The authors thank Daniel Herrmann and his team from the Orthopedic and Rehabilitation Engineering Dresden, Dresden, Germany for the production and help during the advancement of the silicone finger cap.
